# A Model for Evolutionary Structural Plasticity and Synchronization of a Network of Neurons

**DOI:** 10.1155/2021/9956319

**Published:** 2021-06-16

**Authors:** Gualberto Solís-Perales, Jairo Sánchez Estrada

**Affiliations:** Depto. de Electrónica, CUCEI, Universidad de Guadalajara, Av. Revolución No. 1500, Guadalajara, Jal. C.P. 44430, Mexico

## Abstract

A model of time-dependent structural plasticity for the synchronization of neuron networks is presented. It is known that synchronized oscillations reproduce structured communities, and this synchronization is transient since it can be enhanced or suppressed, and the proposed model reproduces this characteristic. The evolutionary behavior of the couplings is comparable to those of a network of biological neurons. In the structural network, the physical connections of axons and dendrites between neurons are modeled, and the evolution in the connections depends on the neurons' potential. Moreover, it is shown that the coupling force's function behaves as an adaptive controller that leads the neurons in the network to synchronization. The change in the node's degree shows that the network exhibits time-dependent structural plasticity, achieved through the evolutionary or adaptive change of the coupling force between the nodes. The coupling force function is based on the computed magnitude of the membrane potential deviations with its neighbors and a threshold that determines the neuron's connections. These rule the functional network structure along the time.

## 1. Introduction

The human brain comprises approximately 10^11^ neurons, which have 10^15^ physical connections between them [1]. Such a network's inherent complexity has made it difficult to decipher the principles by which the brain can be synchronized and perform complex tasks. This issue has induced the study of the brain using the theory of synchronization in complex networks. The synchronization and the interaction of some regions in the brain are a challenging problem. Gabriele Arnulfo and coworkers [2] reported experimental evidence that phase synchronization of high-frequency oscillations reproduces structured communities. This synchronization is transient since it can be enhanced or suppressed. It is known that synchronization in some sense (phase synchronization, complete synchronization, generalized synchronization, lag synchronization) is the mechanism through which the brain regions are integrated. This synchronization between brain regions or some group of neurons can appear at different times. In different regions or neurons, neurons or groups of neurons can participate in different groups at different times [3].

Synchronization is a phenomenon that occurs when units of a set interact dynamically and adjust some of their properties to arrive at simultaneity in time. It is intrinsic, from the highest levels of organization: the world economy, the stock market, and ecological systems [4–6] down to the lowest levels: chemical reactions, circadian rhythms, and neurons in the brain [7–9]. It is not surprising that nature produces an organization to achieve the synchronization of its processes. If it is assumed that everything in the universe is connected, in a network, then it incites to think that there is some pattern of synchronization. That is the main reason why the study of the network's synchronization is fundamental. The scientific development of the synchronization theory, from the first advances made by Winfree and Kuramoto [10, 11] to the latest research, has reduced the problem of scientifically describing the phenomenon for each particular network to simply studying the topology of different networks [12–16].

From the moment when oscillatory responses were discovered in the visual cortex of cats and between areas of the human brain [17–19], the study of the dynamics of neurons as a whole has been focused on the synchronization of complex networks as a viable way in understanding the cognitive function of the brain [1, 20]. Between different networks, there are the structural network and the functional network. Bressler [20] defines the structural network as a set of interconnected neural units, anatomical connections in white matter (axonal fibers) that join different brain regions. Also, Bressler defines the functional network as a collection of interconnected areas of the brain that interact to develop a function [20]. The significant advances suggest that the brain's cognitive functions depend on the activity and coactivity of large populations of neurons in distributed networks [1], among other discoveries.

Models of neural networks have been proposed to elucidate the interaction's laws between regions of the brain's functional networks, using synchronization theory. Such models have included characteristics and topological properties of the brain network, and they have shown that they could reach synchronization. For example, Kuramoto's generalized model has helped to describe how frequencies and synaptic plasticity affect the synchronization of the neural network in a more realistic way [21]. Nevertheless, the disadvantage is that each neuron is characterized as an oscillator, which leaves aside the wide range of dynamic behaviors that the neuron could present [22]. There is also evidence that the brain's structural and functional networks have the properties of small world and modularity [23–25]. In these works, a weaker form of synchronization was found, called phase synchronization. It was also found how the neurons, characterized by the Rulkov or Huber-Braun model, produce an oscillatory behavior capable of synchronizing at different phase values under certain coupling conditions, which reduces the system to a Kuramoto model. The proposed neural network models can give an idea of how the different parts of the brain perform tasks as a whole. However, these models only produce a fixed functional network that does not model the results found experimentally [26].

In the study of the brain, one of the goals is to find out how the structural network, relatively fixed, produces the functional network's evolutive patterns at the same time reaches synchronization [26]. Experiments have shown that the functional connections' patterns and coupling forces may change according to the tasks demanded. For this reason, it is not enough to model a structural network with fixed couplings or time-dependent structural plasticity for all connections since the generated functional network will be fixed. In [27], Yan proposed a rule that governs the interconnection forces of the network. He also suggested that the coupling is a function of the error. The coupling force between neurons grows as more discrepancy is found in their behaviors, allowing the network to reach synchronization. Yan's work shows an advance concerning previous results since he has suggested a variable coupling depending on the error. Such a premise leads the neuron network to a fixed connection, which means that the coupling reaches a fixed value and generates a fixed functional network. To be specific, the so called obtained evolution is only a change in the coupling value. Therefore, it cannot be considered an evolution of the network's structure.

In this work, we propose a model that reproduces the evolutionary dynamics of a functional network of neurons from a fixed structural network. It is essential to mention that there are several possible terms within the category of temporal networks to name these models [28]. However, mainly, there are two of them: the time-varying networks, where the changes in the network properties are purely dependent on time, and the nodes' behavior does not change the network's properties. In contrast, state-dependent networks are such that the nodes' behavior can modify the network's characteristics. Thus, the model proposed here depends on the neurons' membrane potential. This model is considered a temporal network; however, as the model depends on the neuron's states, the proposed model is state-dependant. The level of the membrane potential defines the evolution. In this way, the connected neurons contribute to their connections, whereas some other neurons reduce the coupling strength to form some communities or groups of neurons. Each neuron dynamic is the Hodgkin-Huxley model [29]. The rule that dictates the topology of the functional network and the coupling force between neurons is a function that depends on the state of the network elements. The model allows the generation of a synchronizable functional network, whose configuration in the connections evolves according to the neurons' membrane potential affinity. The model generates clusters of neurons with similar transient synchronous behavior. Also, the network is reorganizing and forming new clusters. The neurons via the evolutionary couplings define the evolution of the network structure so that over time, there are clusters of formation or related neurons' communities. Coupling force is taken from a model that describes particles' movement in gases [30], where their positions are determined by their neighbors and the distance between them. In such a way, some particles influence other positions as long as they are within a spatial range. In this work, this idea is taken for modeling the synchronization of a network of neurons, which describes evolutionary behavior in the interconnection of neurons or neurons' groups.

## 2. Evolutionary Network Model of Neurons

A system composed by *N* interconnected dynamic units can be represented by a network. The equations of a network are described by

(1) $$\begin{array}{c} {\dot{x}}_{i}=f\left(x_{i}\right)+c_{i}\overset{N}{\underset{j=1}{\sum }}a_{ij}\Gamma x_{j},i=1,2,\cdots ,N. \end{array}$$

In the model, **x**_*i*_ = (*x*_*i*1_, *x*_*i*2_,⋯,*x*_in_)^*T*^ ∈ **R**^*n*^ is the state variables of the *i*-th node, *f*(**x**_*i*_): **R**^*n*^ → **R**^*n*^ is a real-valued vector field of the system in the node, *c*_*i*_ represents the coupling strength, and Γ ∈ **R**^*n*×*n*^ is the inner coupling constant matrix that links coupled variables between nodes. This matrix Γ defines through which state that the connection with other neurons is made. In this case, the interaction between neurons is modeled through the injection of currents. The network Laplacian matrix *A* = (*a*_*ij*_) ∈ **R**^*N*×*N*^ represents the scale and topology of the network. The Laplacian matrix satisfies *A* = (*a*_*ij*_) = *𝒜* − *D* with *𝒜* the coupling matrix and *D* the diagonal degree matrix. If there is a connection between the *i*th and *j*th nodes, then *a*_*ij*_ = 1. Otherwise, if there is no connection, then *a*_*ij*_ = 0, the diagonal elements *a*_*ii*_ = −*k*_*i*_ with *k*_*i*_ the degree of the node *i*. In Eq. (1), excitatory and inhibitory neurons can be considered. In this work, only excitatory neurons are taking into account. It is not straightforward to prove the stability of networks containing inhibitory neurons.

Each node dynamics is represented by a neuron dynamics using the Hodgkin-Huxley model [29]:

(2) $$\begin{array}{c} C_{M}\dot{V}=-I_{Na}\left(t\right)-I_{K}\left(t\right)-I_{L}\left(t\right)+I\left(t\right)=-g_{Na}m^{3}h\left(V-E_{Na}\right)-g_{K}n^{4}\left(V-E_{K}\right)-g_{L}\left(V-E_{L}\right)+I\left(t\right)\dot{n}=\alpha_{n}\left(V\right)\left(1-n\right)-\beta_{n}\left(V\right)n,\\ \dot{m}=\alpha_{m}\left(V\right)\left(1-m\right)-\beta_{m}\left(V\right)m,\\ \dot{h}=\alpha_{h}\left(V\right)\left(1-h\right)-\beta_{h}\left(V\right)h. \end{array}$$

The first state variable is the membrane potential *V* whose time derivative is proportional to the sum of the ionic currents flowing through the neuron's membrane. The three remaining state variables *n*, *m*, and *h* model the probability that an ion channel is open at a given moment. *I*_*Na*_(*t*), *I*_*K*_(*t*), *I*_*L*_(*t*), and *I*(*t*) represent the electric currents produced by the ionic currents of sodium, potassium, and chloride, respectively, and the currents injected externally. *E*_*Na*_, *E*_*K*_, and *E*_*L*_ are the equilibrium potentials for sodium, potassium ions, and the potential of the zero leakage current due to chloride ions and others. The constants *g*_*Na*_, *g*_*K*_, and *g*_*L*_, represent the maximum conductance. *α*_*n*_(*V*), *β*_*n*_(*V*), *α*_*m*_(*V*), *β*_*m*_(*V*), *α*_*h*_(*V*), and *β*_*h*_(*V*) express rates of change which vary with voltage but not with time.

The network synchronization of neurons means synchronization in the membrane potential. Therefore, the *i*th node's interconnection, in the right part of Eq. (1), is carried out through the first state variable of Eq. (2).

The concept of evolution in a network leads us to think that it is necessary to change the topology derived from the nodes' dynamic interaction. In other words, it means that the network matrix *A* is a function of the state variables of the neurons. Therefore, to have a functional evolutionary network of neurons that models the various functional network patterns observed in the brain and generated under a fixed structural network, the network matrix must be a function of the membrane potential which this is *A*(*V*(*t*)) and *a*_*ij*_(*V*). Then, the problem is to find a rule that dictates which nodes will be connected and why.

In this work, a vector and a matrix used in coupled maps are proposed, which models coupled dynamic systems whose couplings change depending on the system elements' state variables and their interactions [31].

(3) $$\begin{array}{c} r_{i}=r_{0i}+\underset{j\in \eta_{i}}{\sum }\frac{r_{0j}-r_{0i}}{\left|r_{0j}-r_{0i}\right|}F\left(x_{j},x_{i}\right), \end{array}$$

(4) $$\begin{array}{c} A\left(r\right)=\left(\begin{array}{cc} a_{ij}=1, & \left|r_{j}-r_{i}\right|\leq R,\\ a_{ij}=0, & \left|r_{j}-r_{i}\right|>R. \end{array}\right. \end{array}$$

The vector *r*_*i*_ indicates the position of the *i*th neuron, at the next time instant, of the neuron connections in a *d*-dimensional space. The vector *r*_0*i*_ is the position in the current time of the *i*th neuron and provides the direction and sense of the connection. In Eq. (3), the set of elements interacting with the *i*th element is denoted by *η*_*i*_ = {*j* : |*r*_0*j*_ − *r*_0*i*_| ≤ *R*}. The number of elements in *η*_*i*_ is *N*_*η*_*i*__. *F*(*x*_*i*_, *x*_*j*_) is a function that provides an attraction or repulsion that depends on the state of the *i*th and *j*th element. This function determines the sense of the connection. The *N* elements of the system are placed in a spatial region [*L*_0_, *L*_*f*_]^*d*^ of dimension *d* with periodic boundary conditions, where *L*_0_ and *L*_*f*_ are positive parameters that define region's size. Such a vector, in a coupled map, allows to model social behaviors of communities in social-ecological competition [30]. When introduced as social rule in the neuron model, it is useful to approximate an answer of one of the critical questions about cognition: how the different functional networks cooperate, compete, and coordinate their activity during complex cognitive behavior? [20]. Therefore, in our model, the vector in Eq. (3) will determine where the *i*th neuron will send its information. In this way, the network matrix *A*(*r*(*x*)) of the functional network is a function of the system state variables and models the formation and destruction of synaptic connections between neurons. These functions (3) and (4) model or define the synaptic plasticity by the variation of the conductance in the electrical synapse since the conductance determines the neuron coupling [32].

The structural network characterizes the physical wiring. In other words, it is the network that describes the configuration of the axonal and dendritic connections between neurons. Then, in our model, this network is specified as a set of spatial regions [*L*_0*i*_, *L*_*fi*_]^*d*_*i*_^ of dimension *d*_*i*_ with periodic boundary conditions on a periodic plane [*L*_0_, *L*_*f*_]^*d*^. Each periodic space [*L*_0*i*_, *L*_*fi*_]^*d*_*i*_^ restricts the domain of the vector *r*_*i*_ (3) of the *i*th neuron. The geometric centers of the periodic spaces [*L*_0*i*_, *L*_*fi*_]^*d*_*i*_^ represent the structural network and the overlaps between them the connections, see Figure 1. In this way, any structural network can be represented by placing the periodic spaces so that the overlaps between them generate the desired network configuration. Figure 1 shows a neural network of 10 pyramidal neurons, Figure 1(a), represented by ten planes of a different color, Figure 1(b). Each plane represents the branching of the axons and dendrites of each neuron (node), while the overlap between one plane and the other means that two neurons are physically connected (edge) because their branches intersect. The numbered planes, Figure 1(c), that represent the branches of the neurons (nodes) correspond to the periodic spatial regions [*L*_01_, *L*_*f*1_]^*d*_1_^, [*L*_02_, *L*_*f*2_]^*d*_2_^, ⋯, [*L*_010_, *L*_*f*10_]^*d*_10_^, which restrict the displacement of the vectors *r*_1_, *r*_2_, ⋯, *r*_10_, respectively. If any neuron of the physical network of Figure 1(a) and the plane corresponding to that neuron in Figure 1(b) is analyzed, it will be realized that there is a correspondence between the neurons' connections with its neighbors and the overlaps between the plane with neighboring planes, Figure 1(c). For example, in Figure 1(a), neuron *G* is connected to neuron {*D*, *B*, *A*^2^}, and plane 7, representing neuron *G*, overlaps with planes {4, 2, 10}, representing neurons {*D*, *B*, *A*^2^}.

The proposed model of the functional evolutionary network of neurons, generated under a fixed structural network, is:

(5) $$\begin{array}{c} {\dot{x}}_{i}=f\left(x_{i}\right)+\overset{N}{\underset{j=1}{\sum }}c\left(r_{i},r_{j}\right)a_{ij}\left(r_{i},r_{j}\right)\Gamma x_{j},\\ r_{i}=r_{0i}+\gamma \left(\underset{j\in \eta_{i}}{\sum }\frac{r_{0j}-r_{0i}}{\left|r_{0j}-r_{0i}\right|}\right)\left(\Gamma x_{i}\underset{j\in \eta_{i}}{\sum }\Gamma x_{j}\right),\\ r_{i}\in {\left[L_{0i},L_{fi}\right]}^{d},\;i=1,2,\cdots ,N\in R. \end{array}$$

The function *F*(*x*_*i*_, *x*_*j*_) of the vector at (3) was modified in (5) by Γ*x*_*i*_∑_*j*∈*η*_*i*__‍Γ*x*_*j*_; note that the sign and the magnitude of the states Γ*x*_*i*_ and Γ*x*_*j*_ determine the vector *r*_*i*_'s sense, which means that there is repulsion or attraction between neurons. This new expression generates the sense of the information's movement and can be interpreted as the *i*th neuron's affinity to share information with its neighbor. The parameter *γ* is a gain, and if its value is too large, groups cannot be formed because the change |*r*_0*j*_ − *r*_0*i*_| will be greater than *R*. The coupling force *c*(*r*_*i*_, *r*_*j*_) = *ε*/*N*_*η*_*i*__ with *ε*, a positive constant, indirectly depends on the state. After all, it is necessary to know the vectors *r*_*i*_ and *r*_*j*_. The vectors depend on the state **x** to compute the number *N*_*η*_*i*__ of elements neighboring the *i*th element. The outer coupling *a*_*ij*_(*r*_*i*_, *r*_*j*_) represents the connection between node *i*th and *j*th and is given in (4). It takes values 0 or 1 and is defined by the value of the vector *r* in second equation of (5); thus, *a*_*ij*_(*r*_*i*_, *r*_*j*_) determines if there is or not connection between two neurons according to the value of the function *r*. The coupling strength *c*(*r*_*i*_, *r*_*j*_) also depends on the value of the function **r**, and its value increases or decreases the connection strength between the connected neurons. The proposed model is based on the rules of connections presented in [31], where all the vectors *r*_*i*_ s evolve into a single defined periodic region. We take advantage of this fact, but we modified it, restricting the periodic regions for each *r*_*i*_, allowing us to relate neurons' physical space with the restricted periodic regions of (5). In this way, we modeled the structural network. The functional neuron network is modeled with the first equation of (5). It has an evolutive behavior because the network matrix (4) evolves according to the *r*_*i*_ vectors' movement in its restricted domains. The functional evolutionary network of neurons has the characteristic of connecting and disconnecting in such a way that it generates communities of connected and related neurons. In (5), such behavior is reproduced by the functions (4) and (3) that consider the neurons' potential and increases the coupling strength between neurons if their potentials have the same sign. The previous function leads to neurons grouping with similar or equal neuron's potentials; simultaneously, the spatial regions' restriction forms a fixed structural network [*L*_0*i*_, *L*_*fi*_]^*d*^.

## 3. Evolution and Synchronization of the Network Neurons

The objective of a controller is to force the error system to converge to zero and to be able to obtain outputs similar to the input reference. If the complex network's model (1) is analyzed, it can be concluded that the term *c*∑_*j*=1_^*N*^‍*a*_*ij*_Γ**x**_*j*_ forms a controller that forces the dynamics of the elements to be the same over time. Synchronization of the elements is then achieved if the controller can drive the error system to zero.

Assuming *N* isolated elements, where the dynamics of the *i*th element are given by

(6) $$\begin{array}{c} {\dot{x}}_{i}=f\left(x_{i}\right),i=1,2,\cdots ,N, \end{array}$$

then the error dynamic is

(7) $$\begin{array}{c} e_{i}=\overset{N}{\underset{j=1}{\sum }}\left(x_{i}-x_{j}\right),i=1,2,\cdots ,N. \end{array}$$

Up to this point, the system is in open loop. Now, if the *N* isolated elements of the system (6) are coupled by some of their states, then the error will be

(8) $$\begin{array}{c} e_{i}=\overset{N}{\underset{j=1}{\sum }}a_{ij}\Gamma x_{j},,i=1,2,\cdots ,N, \end{array}$$

where *a*_*ij*_ ∈ **R**^*N*×*N*^ provides the outer configuration of how the *N* elements are coupled, and Γ ∈ **R**^*n*×*n*^ is a constant matrix with values of 0 or 1 that links inner coupled variables. The element ∑_*j*=1_^*N*^‍*a*_*ij*_*x*_*j*_ lumps the error (7), because *a*_*ii*_ = −*k*_*i*_. If the error is multiplied by a gain *c*, then there is the same form (1). The Eq. (8) can be seen as a proportional controller that tries to drive the *N* elements' system to synchronization. The isolated dynamics of the *N* elements, plus the proportional controller, is called a complex network.

If the right-hand side of the first equation in (5) is analyzed, it can be observed that it forms an adaptive controller for network synchronization. The sum represents the error, which are the differences between the *i*th neuron's action potential and the *j*th neighboring neuron. The adaptive gain of the controller is the function of the coupling strength *c*(*r*_*i*_, *r*_*j*_). The outer coupling *a*_*ij*_ depends on the vector (3) and model whether there is an exchange of information between neurons, favoring evolution in the functional network. Then, the evolution is given by the adaptive coupling strength. Simultaneously, the structural network is fixed with the topology dictated by the geometric position of the periodic domains [*L*_0*i*_, *L*_*fi*_]^*d*^ in the periodic plane [*L*_0_, *L*_*f*_]^*d*^.

In order for a network with a fixed configuration to reach synchronization, it is enough to show that the error system converges to zero, as was reported in [12, 34]. In this works, the synchronization is achieved in an isolated node $\dot{\mu }\left(t\right)=f\left(\mu \left(t\right)\right)$. The solution *μ*(*t*) can be an equilibrium point, a periodic orbit, or a chaotic attractor. In our work, apart from proving the synchronization in the complete network, it is also considered the difference between synchronized neurons' average and the neuron potential as a synchronization level [35]. Due to the network matrix evolutionary behavior (4), the network configuration is changing over time. Although evolutionary behavior impedes to prove synchronization for all the time, the network's synchronization can be proved in the intervals where the topology is fixed. In these intervals, the synchronization of (5) can be proved if the network satisfies the necessary conditions reported in [12, 34], where networks with time-varying couplings reach synchronization, as long as the following inequality holds:

(9) $$\begin{array}{c} {\left[Df\left(\mu \left(t\right)\right)+d\Gamma \right]}^{T}G+G\left[Df\left(\mu \left(t\right)\right)+d\Gamma \right]\leq -\sigma I_{n} \end{array}$$

for all $d\leq \bar{d}<0$ and $\lambda_{2,\max}\leq \bar{d}<0$, where *Df*(*μ*(*t*)) is the Jacobian matrix at the isolated solution, and *λ*_2,max_ is the largest eigenvalue of the network. If the inequality is satisfied, then it means that there exists a spanning tree in the network. Then, the synchronization between the neurons is achieved with $\bar{d}<0$ that is a constant value that ensures exponential synchronization. The inequality (9) is used to determine whether the synchronization between neurons' potentials is exponential. The condition is satisfied if the second largest eigenvalue of the network matrix is less than a constant parameter $\bar{d}<0$ less than 0. These necessary conditions for synchronization were reported in 2002 by Chen in [12, 16] and were used in [34], with time-varying coupling networks. The network topology is changing due to the couplings' evolutionary behavior between nodes in the functional network. Therefore, the stability can be ensured in time intervals where there is a fixed topology. Nevertheless, not for the moment when there is a change in a configuration from one network to another. However, it is possible to use the results reported in [34] for time intervals where the network matrix (4) is fixed.

The value for the parameter *d* in Eq. (9) is obtained so that the matrix of the inequality is negative definite. For computing (9), matrix *G* is considered as an identity matrix *I*_4_, for simplicity. The negative definite matrix can be obtained using Sylvester's criterion, which states that matrix Ψ = [*Df*(*μ*(*t*)) + *d*Γ]^*T*^*G* + *G*[*Df*(*μ*(*t*)) + *d*Γ] is negative definite if and only if (−1)^1^Δ_1_ > 0, (−1)^2^Δ_2_ > 0, ⋯, and (−1)^*n*^Δ_*n*_ > 0 with Δ_*k*_ = det(Ψ(*k*)), being Ψ(*k*) the leading principal submatrix of order k. Therefore, each of these equations obtained from the leading principal minors are solved for the parameter *d*. The value of *d* was found as −15209237, which indicates that $\bar{d}$ can be any value close to 0 and then $\lambda_{2,\text{m}a\text{x}}\leq \bar{d}<0$.

(10) $$\begin{array}{c} \psi_{11}=2d-\frac{2\left(g_{Na}hm^{3}+g_{K}n^{4}+g_{L}\right)}{C_{M}},\\ \psi_{12}=\psi_{21}=\frac{0.01n-0.01}{e^{\left(1-V/10\right)}-1}+\frac{0.0016n}{e^{V/80}}+\frac{4g_{K}n^{3}\left(E_{K}-V\right)}{C_{M}}+\frac{0.001e^{\left(1-V/10\right)}\left(V-10\right)\left(n-1\right)}{{\left(e^{\left(1-V/10\right)}-1\right)}^{2}},\\ \psi_{13}=\psi_{31}=\frac{0.1m-0.1}{e^{\left(5/2-V/10\right)}-1}+\frac{0.22m}{e^{V/18}}+\frac{0.001e^{\left(5/2-V/10\right)}\left(m-1\right)\left(V-25\right)}{{\left(e^{\left(5/2-V/10\right)}-1\right)}^{2}}+\frac{3g_{Na}m^{2}h\left(E_{Na}-V\right)}{C_{M}},\\ \psi_{14}=\psi_{41}=\frac{0.0035h-0.0035}{e^{V/20}}+\frac{g_{Na}m^{3}\left(E_{Na}-V\right)}{C_{M}}-\frac{0.01e^{\left(3-V/10\right)}h}{{\left(e^{\left(3-V/10\right)}+1\right)}^{2}},\\ \psi_{22}=\frac{2\left(0.01V-0.1\right)}{e^{\left(1-V/10\right)}-1}-\frac{0.25}{e^{V/80}},\\ \psi_{23}=\psi_{32}=0,\\ \psi_{24}=\psi_{42}=0,\\ \psi_{33}=\frac{2\left(0.01V-2.5\right)}{e^{\left(5/2-V/10\right)}-1}-\frac{8}{e^{V/18}},\\ \psi_{34}=\psi_{43}=0,\\ \psi_{44}=-\frac{0.14}{e^{V/20}}-\frac{2}{e^{\left(3-V/18\right)}+1}. \end{array}$$

The elements *ψ*_*ij*_ of the matrix Ψ = *ψ*_*ij*_ of the functional network calculated for the instant of time [*t*_0_, *t*_1_] are in (10). Equation (9) is used to prove that exponential synchronization can be reached in each interval [*t*_0_, *t*_1_] where the topology is fixed. However, it is not known what the synchronization level of the network is, if all neurons are synchronized with the same magnitude or if there are neurons that are more synchronized with one another.

To analyze the synchronization level of the connected neurons, a measure of the synchronization is desirable. A synchronization measure of the synchronized neurons in a network or a specific community can be defined as the logarithm of the standard deviation of the membrane potential over the network (or community) and the average of the network's potentials (or community's potentials). Consider the average of the states (membrane potential) in the time interval [*t*_0_, *t*_1_] as

(11) $$\begin{array}{c} \mu \left(t\right)=\frac{1}{N}\overset{N}{\underset{i=1}{\sum }}\Gamma x_{i}\left(t\right)=\frac{1}{N}\overset{N}{\underset{i=1}{\sum }}V_{i}\left(t\right). \end{array}$$

Now, the standard deviation is calculated as

(12) $$\begin{array}{c} \sigma \left(t\right)=\sqrt{\frac{1}{N}\overset{N}{\underset{i=1}{\sum }}{\left(\Gamma x_{i}\left(t\right)-\mu \left(t\right)\right)}^{2},} \end{array}$$

and the synchronization level measure (synchronization index) is calculated as follows:

(13) $$\begin{array}{c} S\left(t\right)=-\ln\left(\sigma \left(t\right)\right). \end{array}$$

If the synchronization index *𝕊*(*t*) is positive, then the neurons' membrane potential is close enough, and the synchronization between nodes is reached [35].

One of the fundamental behaviors produced by model (5) is that it produces different clusters of highly connected neurons over time, defined as communities. For this reason, it is necessary to use an algorithm that identifies and determines the number of communities formed at the instant of time where the functional network has a fixed topology. In this work, an algorithm based on modularity optimization is used to detect the communities at every moment [35]. It is essential to note that the detection of communities in any network does not depend on synchronization between nodes. In the opposite direction, synchronization between nodes does not depend on communities. It is only necessary to analyze the matrix of external links *A* = (*a*_*ij*_), representing the network topology, to perform communities' detection.

In this way, once the communities are detected, the index (13) can be calculated for the functional network and for the communities formed within the network. In this way, it is possible to know if the neurons that belong to the same community exhibit a greater synchronization index than those that do not belong to the community. As the network topology is evolving, therefore, a node can belong to different communities over time. The probability that two different neurons belong to the same group is calculated all time to solve this issue. If two neurons meet a 70% probability of belonging to the same group, the neurons are said to belong to the same community.

### 3.1. Simulation Results

The numerical simulation of the model was carried out with the values of the parameters given in Table 1. The numerical integration of the model was performed with the Matlab integration ODE45 function. This function implements a Runge-Kutta method with the Dormand-Prince pair variable time step for efficient computation. Model (5) was simulated over 3000 milliseconds. From time 0 to less than 400, the neurons were simulated without connection between them. In Figure 2, there were only isolated neurons. It is important to note that isolated neurons have different behaviors between them. From time 400 to 3000, the neurons were simulated as a network. Sixty-four neurons were used due to processing capacity issues since the Hodgkin-Huxley model used for each node requires many iterations to perform its numerical integration. It is possible to generate a network with any number of nodes, but it will depend on the processing capacity.

The structural network used in the simulation was a lattice network. All the neurons' dendrites and axons were connected. Evolution exists when there are different configurations of the network over time, and the coupling function depends on some state of the system. Therefore, for the proposed model (5), the change of the node degree ensures evolution.

The evolution of the functional network obtained in the simulation is shown in Figure 3. As the graphic is traversed, at a fixed height, from the vertical direction through the horizontal direction, there is a color change indicating the degree variation of the node. The change in color in the horizontal direction, from time 400 to 3000, ensures a change in the network configuration over time, and that the node's degree is different from its neighbors.

It is essential to highlight that although the network's topology is evolving concerning the state, it reaches a synchronization in the neurons' membrane potentials, as Figure 2 exhibits. The intensity of color represents the magnitude of the potential, whose unit is the millivolt, and the voltage goes from -100 mV to 40 mV, which is lower than the resting potential of 50 mV. Figure 2 shows how the 64 neurons synchronize their action potential one time they are not isolated. If the graph is traversed vertically, there is no change in the color intensity, which shows that the neurons reached a simultaneity in their voltages from time 400 to 3000.

Figure 4 shows the largest eigenvalue *λ*_2,max_ < 0 of the network matrix (4), where despite the evolution in the connections, the network synchronizes in the time interval *T*_*S*_ = [400, 3000].

In Figure 5, the synchronization index *𝕊*(*t*) is changing due to the evolutionary characteristic of the network. Notice that for some time intervals, for instance, *T*_1_ = [1400, 1450], the synchronization index *𝕊*(*t*) is negative, which means that the synchronization is weak. On the other hand, the synchronization index is positive and has a maximal value in the time intervals *T*_2_ = [400,450], *T*_3_ = [700,750], and *T*_4_ = [1800, 1850]. On the intervals for the spikes, the synchronization index changes due to the membrane potential variation; however, synchronization is sustained. It is important to stress that if the synchronization index is positive, then the standard deviation is less than 1, and the behavior of the membrane potentials is very close each other, whereas if it is negative, it only means that the membrane potentials are weakly synchronized, but the qualitative behavior remains. The synchronization of the membrane potential is illustrated in Figure 2, where it can be seen the synchronization of the spikes around *t* = 1000 msec. and *t* = 2500 msec. Each vertical line corresponds to one spike in each neuron.

Moreover, the coupling evolutionary model and the synchronization criteria generate communities of neurons with similar synchronous behavior. The algorithm reported in [36] was used to compute the detection of communities that the proposed network can form over time and observe they are changing.  Figure 6 shows the change at each time in the number and size of the communities formed in the network. As the graphic is traversed horizontally, different numbers of communities can be found over time, proving emergence or dissolution of communities. Also, there is a color intensity change at each time, indicating the of the size communities. This graph shows that there exist groups of neurons densely connected.

Suppose a group of neurons in a network is very connected, in that case, the neurons have more probabilities of exhibiting similar behaviors because the connections work as controllers that force the neurons to reach synchronization. To illustrate by means of simulation this previous idea in simulation, based on identifying the neurons that belong to each community formed over time, from 400 to 3000, each neuron probability membership to each community formed is computed. Neurons that belong with more than 70% of probability to the same community over all the time are in Figure 7. This figure shows the computed index (13) for each of the more probable communities from 400 msec to 3000 msec. The index for the communities in Figure 7 shows that the neurons that belong with more probability to the same group exhibit strong synchronization because the index has a positive value the major part of the time. This result contrasts with the result that exhibits in Figure 5, where all the neurons in the functional network display weak synchronization the major part of the time. Therefore, it shows that the proposed model generates communities of neurons with synchronous behaviors.

## 4. Conclusions

The result shows the evolutionary synchronization of a network of neurons. Evolution is understood as the change in the functional network structure in terms of the connected neurons' potentials, those neurons whose membrane potential is close. Then, the proposed model generates a class of evolutionary patterns in the functional network of neurons. This evolutionary behavior represents the attenuation or increment of the electrical connection between neurons. Similar behavior has been observed experimentally in living beings. The coupling between neurons can be seen as an adaptive controller that forces the network to converge to practical synchronization between subgroups of neurons, even as the couplings matrix evolves. The coupling matrix, being dependent on the membrane potential through a function that reproduces social behaviors, generates changes in the topology, which is purely defined by the connections between neurons at a particular time. Furthermore, the affinity between the potentials of neurons with synchronous behavior sets the guideline for such connections. Finally, there was a finding that different subgroups of neurons with different behaviors can be generated in the same network. This phenomenon can be understood as executing different tasks performed by the same network of neurons, where each task can be seen as a particular synchronous behavior. Even though it is a simplified model of the human connectome, the results in this work can be extended to larger dimensions. Each periodic region proposed in the model representing the neuron's space can be whichever topological manifold. Thus, there exist manifolds that correctly model the neuron's space of whichever structural network.

## Figures and Tables

**Figure 1:** The construction process of the structural network, using the domains [*L*_0*i*_, *L*_*fi*_]^*d*_*i*_^ that restrict the motion of the vector (3) for each neuron, from a real network of neurons. (a) Pyramidal cells: they are characteristic of the olfactory cortex of man, resident in the piriform lobe, and the hippocampal gyrus, Ramon y Cajal [33]. (b) Representation of the neural ramification and its connections, in the structural network, through the spatial periodic domains and their overlaps. (c) The resulting structural network modeled using the overlap (links) of the domains (numbered nodes).

**Figure 2:** Network synchronization. The *Y*-axis represents the 64 nodes' index of the network, the *X*-axis represents time, and each color of the right bar represents the membrane potential with mV. The vertically constant intensity of color on the graph, over time from time 400 to 3000, shows that there is synchronization in the membrane potentials of the neurons. There is no synchronization from 0 to less than 400 because neurons are isolated like the change of color shown on the graph.

**Figure 3:** Evolution of the functional network. The *Y*-axis represents the 64 node's index of the network, the *X*-axis represents time, and each color of the right bar represents the number of neighbors connected to the node. The variation of color intensity when moving horizontally on the graph shows the evolution of the network. From time 0 to less than 400, there is no evolution. Colors are constant horizontally because neurons are isolated, but from time 400, the neurons are connected, and there is a change of color; thus, there is evolution.

**Figure 4:** The maximal eigenvalue *λ*_2,max_ of the network in each period where the network matrix is constant. There is *λ*_2,max_ = 0 from time 0 to less than 400 because neurons are isolated, and then it means that there is no spanning tree in the network. From time 400 to 3000, there is a spanning tree in the network because the neurons are connected, and so the largest eigenvalue *λ*_2,max_ is calculated. It is essential to see that from time 400 to 3000, the largest eigenvalue is always negative.

**Figure 5:** Mean value of the neuron potential (11) (black signal) between the 64 neuronal behavior (blue signal). The first graph shows how the 64 neurons' behavior is close to the mean value, while the second graph confirms this synchronization through the index's positive values *𝕊*(*t*) of the functional network.

**Figure 6:** Community detection in the neural network. The *Y*-axis represents the community's index in the network, the *X*-axis represents time, and each color of the right bar represents the numbers of neurons belonging to each community. The color's change over time shows how the amount and size of the communities are changing, proving that there can be the forming and destroying communities.

**Figure 7:** Index's values *𝕊*(*t*) of the probable neuron communities formed in the functional network over time. The graphs show through the index's positive values *𝕊*(*t*) how the neural behaviors between neurons of the same community are more similar than others which not belong to the same community Figure 5.

**Table 1:** Parameters used in the numerical simulation of the neural network.

Parameter	Value	Parameter	Value
*g*_*Na*_	120 mS/cm^2^	*E*_*Na*_	55 mV
*g*_*K*_	36 mS/cm^2^	*E*_*K*_	-72 m*V*
*g*_*L*_	0.3 mS/cm^2^	*E*_*L*_	-49.4 mV
*C*_*M*_	1 *μ*F/cm^2^	*ε*	18.82
*L*	100	*γ*	6 × 10^−7^
*N*	64	*d*	2
*R*	25		

## Data Availability

All data supporting the results can be found in the manuscript.
